# Mechanism of QingHuaZhiXie Prescription Regulating TLR4-IECs Pathway in the Intervention of Diarrhea Predominant Irritable Bowel Syndrome

**DOI:** 10.1155/2021/5792130

**Published:** 2021-11-09

**Authors:** Hua Huang, Ping Zhao, Meijuan Xi, Fang Li, Lijiang Ji

**Affiliations:** ^1^Department of Anorectal, Changshu Hospital Affiliated to Nanjing University of Chinese Medicine, Changshu 215500, China; ^2^Digestive System Department, Affiliated Hospital of Nanjing University of Chinese Medicine, Nanjing 210000, China

## Abstract

To investigate the effect and mechanism of QingHuaZhiXie prescription on diarrhea predominant irritable bowel syndrome (D-IBS), animal models of rats were used in this study. 48 rats were randomly divided into 6 groups, containing one control group, one animal model group (D-IBS group), and four drug intervention groups (low, medium, and high dosage of QingHuaZhiXie prescription and trimebutine maleate intervention group). Abdominal withdrawal reflex (AWR) and Bristol stool form scale were recorded; the expression levels of inflammatory factors (TNF-*α* and IFN-*γ*), pathway proteins TLR4, MyD88, NF-*κ*B, and key proteins of tight junction between intestinal epithelial cells (IECs) were detected; the microstructure of intestinal mucosal was observed by hematoxylin and eosin (H&E) staining; MPO activity was detected with immunohistochemical analysis to reflect the inflammation of tissues. Results show that QingHuaZhiXie prescription reduced diarrhea index and intestinal hypersensitivity and intestinal tissue integrity after intervention. MPO activity in QingHuaZhiXie prescription-treated rats was significantly lower relative to their model group. The expression levels of inflammatory factors and TLR4/MyD88/NF-*κ*B pathway proteins were repressed, and the protein levels of occludin and claudin-1 increased. Meanwhile, this study also found that the remission effect of QingHuaZhiXie prescription on D-IBS increased with its dosage increase. Hence, as a therapeutic prescription for D-IBS, QingHuaZhiXie prescription could relieve D-IBS symptoms through balancing the inflammatory factors expression by inhibiting the TLR4/MyD88/NF-*κ*B pathway and maintaining the function and structure of IECs by improving the protein levels of JAM, occludin, claudin-1, and ZO-1.

## 1. Introduction

Irritable bowel syndrome (IBS) is one of the most common functional gastrointestinal disorders. The incidence of IBS has reached to 10–30% in the world; furthermore, the incidence is still increasing year by year [1, 2]. According to symptom phenotype, IBS can be divided into four types. Among them, diarrhea predominant IBS (D-IBS) is the most common subtype, which is often accompanied by abdominal distension and watery stool, which has serious impact on patient [2–4].

Numerous factors have been shown to be associate with D-IBS, such as brain-gut axis dysfunction, intestinal flora disorder, intestinal bacterial infection, gastrointestinal motility disorder, visceral hypersensitivity, and so on. However, the pathogenesis of D-IBS is complex, and its pathophysiological mechanism is still unclear [5, 6]. With the research deepening, the importance of the immune inflammatory model in the D-IBS pathogenesis was focused. TLR4 protein belonging to Toll-like receptor family has been recognized as an important element in intestinal inflammatory stress response [7–9]. In response to D-IBS, the TLR4/MyD88/NF-*κ*B pathway, composing of TLR4, myeloid differentiation factor 88 (MyD88), and nuclear factor-*κ*B (NF-*κ*B), can transmit inflammatory signals to inflammatory cytokines such as IFN-*γ* and TNF-*α*, causing imbalanced expression of inflammatory cytokines, leading to inflammatory response, and ultimately affecting gastrointestinal motility, secretion, and sensitivity [5, 7–9].

Dysfunction of intestinal mucosal barrier was observed in D-IBS patient recently [10, 11]. The function of intestinal mucosal barrier is inseparable from the integrity of IECs. Of course, it also includes the junction structure between epithelial cells, which is mainly connected by tight junction (TJ) [12]. TJ is mainly composed of transmembrane proteins, JAM, occluding, and claudin, which form a ring structure at the apical end of epithelial cells. The proteins occludin and claudin, together with zonula occludens (ZO) and other connexins, form junction complexes (JC), whose “zipper like” structure can effectively close the top of the intercellular space and prevent macromolecules invasion [10, 12, 13]. Previous research studies showed that the transcription level of occludin and ZO-1 was significantly repressed in D-IBS patients. Furthermore, the mucosal permeability of D-IBS patients was higher than that of the control group based on the intestinal permeability test [11].

Western medicines have been used in the clinical treatment of D-IBS, such as mesalazine, lalaratide acetate, trimebutine maleate, rifaximin, and bile acid chelator. But the curative effect is relatively simple and often cannot deal with complex D-IBS symptoms [14–16]. Traditional Chinese medicines prescription following the principle of syndrome differentiation and treatment has also been successfully applied in the clinical treatment of functional gastrointestinal diseases [17, 18]. The monomeric components used in traditional Chinese medicine prescriptions for the treatment of IBS include tangerine Radix Paeoniae Alba, Pericarpium Citri Reticulatae, and Fangfeng [17, 18]. On this basis, we further optimized the prescriptions, obtained QingHuaZhiXie prescription, and found that it has a significant effect in the treatment of D-IBS. Furthermore, the animal model of rats was used to elaborate the mechanism of QingHuaZhiXie prescription from the overall effect, intestinal mucosal barrier, ultrastructure and immune inflammatory pathway, and other aspects.

## 2. Methods and Materials

### 2.1. Preparation of QingHuaZhiXie Prescription

Select Fengweicao 10 g, Dijincao 10 g, Psoralea 15 g, Coptis 2 g, Simmering Muxiang 6 g, Ginger 6 g; Radix Paeoniae Alba 15 g, Fangfeng 10 g, Rhizoma Atractylodis 10 g, fried Radix Atractylodis 15 g, and Cranegrass 12 g. All of the medicines were purchased from Beijing TRT Co., Ltd. (Beijing, China). All raw materials in the formula were examined according to the quality control criteria in the Chinese Pharmacopoeia. Take the appropriate amount of each medicinal material, add 10 times the weight of the total medicinal material volume of water, soak 1 h after boiling 1 h, liquid, while hot filtration. The medicinal residue was added with 8-fold volume of water for 1 h, and the filtrate was combined twice to concentrate into 1.2 g/mL medicinal solution. Keep it in the refrigerator at 4°C.

### 2.2. Establishment and Grouping of the Rat Model

The D-IBS rat model was established by neonatal maternal separation (NMS) combined with *Campylobacter jejuni* (ATCC81-176) treatment [19]. 48 rats were randomly divided into 6 groups, containing one control group, one animal model group (D-IBS group), and four drug intervention groups (low, medium, and high dosage of QingHuaZhiXie prescription and trimebutine maleate intervention group). The intervention group of QingHuaZhiXie prescription was given by gavage (low dosage group: 10 mg/kg of twice dilution of crude drug content, medium dosage group: 20 mg/kg, and high dosage group: 30 mg/kg of twice concentration of crude drug), the intervention group of trimebutine maleate was given 15 mg/kg each time (Hainan Puli Pharmaceutical Co., Ltd., China), the D-IBS group was given 10 mg/kg normal saline, while the control group was not treated and intervened.

### 2.3. Intestinal Sensitivity Test

Intestinal sensitivity was assessed by the abdominal withdrawal reflex (AWR) score using the balloon dilator as in a previous research [20]. The AWR score was divided into 0, 1, 2, 3, and 4 scale. The duration of each test was 20 seconds and repeated three times with an interval of 30 seconds.

### 2.4. Stool Form Measurement

Stool form measurement was recorded according to the Bristol stool form scale, ranging from type 1 to type 7 [21]. Feces were collected in metabolic cages from 8: 00 pm. to 8: 00 am. on the next day. During this period, the rats could feed freely.

### 2.5. H&E Staining Analysis

The rats were anesthetized with chloral hydrate as previous report [9]. Colon samples were obtained by dissection and divided into two parts after treatment with normal saline, one for H&E staining and the other for Western blot analysis. The colon tissue about 2 cm was taken out, the intestinal cavity was cut along the mesenteric margin, and the intestinal contents were washed with normal saline, fixed in 4% paraformaldehyde for more than 48 h, washed with distilled water, dehydrated with gradient ethanol, soaked in xylene solution, waxed twice, embedded, sliced, and stained with H&E. The pathological changes of colon were observed under the light microscope.

### 2.6. Western Blotting Analysis

Western blotting analysis was carried out as previous report [9]. Put simply, protein samples of distal colon were extracted by liquid nitrogen grinding and pyrolysis. After the protein concentration was determined by the bicinchoninic acid (BCA) method, 30 *μ*g of protein was taken from each sample and transferred to PVDF membrane (Invitrogen, USA) after electrophoresis. Relative protein levels were detected using corresponding antibodies: TLR4 (AF7017), NF-*κ*B (AF6217), MyD88 (AF5195), occludin (AB216327), and *β*-actin (AF7018) purchased from Affinity (USA) and claudin-1 (AB211737), ZO-1 (AB276131), and JAM (AB52647) purchased from Abcam (USA).

### 2.7. Real-Time Quantitative PCR Analysis

The tissue samples of distal colon were collected from the inferior vena cava. After centrifugation, the sample was collected for the detection of inflammatory factors as previous report [9]. Total RNA was extracted according to RNA extraction kit (ER501-01, TransGen Biotech, China). Real-time quantitative PCR (RT-qPCR) was carried out according to SYBR Green Real-Time PCR MasterMix (AQ602-14, TransGen Biotech, China). The expression level of *β*-actin was used as reference. All primer sequences used in this study are given in Table 1.

### 2.8. ELISA Analysis

The levels of TNF-*α* and IFN-*γ* in serum were detected through ELISA analysis using ELISA kit (Boster, China). The results were calculated according to the instructions and expressed in the concentration of each inflammatory factor (ng/L).

### 2.9. Myeloperoxidase (MPO) Analysis

MPO activities of six groups were detected as previous according to MPO Kit (Nanjing Jiancheng, China) [22].

### 2.10. Statistical Analysis

Statistical analysis was carried out using SPSS 26.0 software. The differences between groups were analyzed by one-way ANOVA, and the least significant difference (LSD) method was used for multiple comparisons. The difference was statistically significant when *P* < 0.05.

## 3. Results

### 3.1. QingHuaZhiXie Prescription Relieves D-IBS Symptoms

The effect of QingHuaZhiXie prescription was analyzed through AWR threshold analysis, stool form measurement, and H&E staining. Reduced AWR pain threshold was observed in D-IBS rats when compared with the control group, while this decreased AWR scale could be rescued by the utilization of QingHuaZhiXie prescription, and the effect was statistically significant (*P* < 0.05). Furthermore, the therapeutic effect of QingHuaZhiXie prescription on D-IBS was positively correlated with its dosage during treatment, and the highest AWR threshold of rats was observed in the high dosage group when compared with that of low and medium dosage (*P* < 0.05) (Figure 1(a)). According to the statistics of fecal characteristics, the Bristol score of the D-IBS model group was higher than that of the control group, but the use of QingHuaZhiXie prescription could effectively reduce the score (*P* < 0.05). Meanwhile, consistent with the results of AWR analysis, the Bristol score of rats in the high-dose group was the lowest in the QingHuaZhiXie prescription intervention group (*P* < 0.05) (Figure 1(b)).

The intestinal epithelium of the control group was complete and orderly, with no loss of epithelial structure and normal glands based on H&E staining result. While, in the D-IBS group, a small amount of inflammatory cells infiltration, submucosal edema, and increased space were observed in the mucosa. Furthermore, degeneration and necrosis of epithelium, separation of epithelium from lamina propria, and damage of part of lamina propria were also found. Although the QingHuaZhiXie prescription intervention group rats also have a small amount of the above phenomenon, it is worth mentioning that both the degree and scope of injury are lighter than the D-IBS group, especially for the rats in the high dosage group of QingHuaZhiXie prescription (Figure 1(c)).

### 3.2. QingHuaZhiXie Prescription Improves the Expression Levels of Occludin, Claudin-1, ZO-1, and JAM

Proteins occludin and claudin-1 are the marker proteins of intestinal mucosal barrier indexes [10, 12, 13]. Western blotting results showed that the expression levels of these two proteins were significantly repressed in the D-IBS model group when compared with that in the control group (*P* < 0.05). However, this repression could be relieved when QingHuaZhiXie prescription was used (*P* < 0.05). With the increase of QingHuaZhiXie prescription dosage, the expression levels of occludin and claudin-1 showed an upregulated trend, and the highest protein expression levels appeared in the high-dose group of QingHuaZhiXie prescription. At this time, the expression level of claudin-1 in the high dosage group had no significant difference from that in the trimebutine maleate group and the control group. Proteins ZO-1 and JAM also play important roles in maintaining the structure and functional integrity of intestinal mucosal barrier. In this study, we found that the expression levels of ZO-1 and JAM were also significantly downregulated in the D-IBS group. After intervention, the expression levels of ZO-1 and JAM proteins in the QingHuaZhiXie prescription group were increased than that in the D-IBS group, and the degree of increase was proportional to the dosage of QingHuaZhiXie prescription. The expression level of internal reference protein *β*-actin was basically the same, indicating that the amount of protein samples was consistent in the experiment, which can eliminate the experimental error (Figure 2).

### 3.3. QingHuaZhiXie Prescription Adjusts the Inflammation Level

The expression levels of inflammatory factors are an important evaluation index of D-IBS [9]. In this study, the effect of QingHuaZhiXie prescription on the expression of TNF-*α* and IFN-*γ* was analyzed by RT-qPCR and ELISA analysis (Figure 3). RT-qPCR results showed that the expression level of TNF-*α* was the highest in the D-IBS model group when compared with the other five groups (*P* < 0.05). While, the transcription level of TNF-*α* decreased with the intervention of QingHuaZhiXie prescription (*P* < 0.05). Meanwhile, with the increase of QingHuaZhiXie prescription dosage, its expression level gradually decreased. Compared with low and medium QingHuaZhiXie prescription dosage groups, the expression level of inflammatory factor TNF-*α* in the high dosage group of QingHuaZhiXie prescription was the lowest (*P* < 0.05). The results of ELISA analysis also showed that the intervention of QingHuaZhiXie prescription could represses the expression level of TNF-*α* (Figure 3(b)). At the same time, it was found that the regulation of proinflammatory factor IFN-*γ* by QingHuaZhiXie prescription treatment was basically consistent with that of TNF-*α* (Figures 4(a) and 4(b)). MPO is an enzyme contained within the granules of neutrophils, and increased MPO activity is associated with severe colitis. Thus, MPO activity is used as a marker of inflammation. MPO activity within the colon of the model group rats was significantly increased compared to that in normal controls (Figure4(c)). However, MPO activity in QingHuaZhiXie prescription-treated rats was significantly lower relative to their model group counterparts. These results further support the colitis-alleviating effect of QingHuaZhiXie prescription.

### 3.4. QingHuaZhiXie Prescription Represses the Expression Levels of TLR4/MyD88/NF-*κ*B

The TLR4-mediated signaling pathway plays an important role in D-IBS, and it is the upstream regulatory unit of inflammatory factor expression [7–9]. In this study, the expression levels of three proteins TLR4, MyD88, and NF-*κ*B in this pathway were detected by RT-qPCR and Western blotting analysis (Figure 3). Results showed that the expression level of TLR4 was the highest in the D-IBS model group, and QingHuaZhiXie prescription decreased the mRNA level of the TLR4 pathway. Compared with the low and medium dosage groups, the high dosage group of QingHuaZhiXie prescription had the highest inhibition (*P* < 0.05). At the same time, the expression level of TLR4 in the high dosage group of QingHuaZhiXie prescription was almost the same with that in the trimebutine maleate group (Figure 3(a)). It should be pointed out that the inhibition of QingHuaZhiXie prescription treatment on TLR4 is not only reflected in the mRNA level but also in the protein level (Figure 3(b)). Similar to the results of TLR4 expression detection, the transcription and translation levels of MyD88 also showed a decreased trend after the intervention of QingHuaZhiXie prescription, and the decreased degree became more obvious with the increase of QingHuaZhiXie prescription dosage (*P* < 0.05). The expression level of NF-*κ*B also showed the same change trend as the former two, that is, it was inhibited by QingHuaZhiXie prescription, and the inhibition degree was the strongest in the high dosage group of QingHuaZhiXie prescription (Figures 3(a) and 3(b)).

## 4. Discussion

As a functional gastrointestinal disease with long duration and easy recurrence, D-IBS seriously affects the quality of life of residents, and its incidence continues to increase. The existing evidence suggests that multiple factors are involved in the occurrence of IBS-D, but its specific and accurate pathogenesis is still unclear. Neonatal maternal separation combined with *Campylobacter jejuni* treatment was used to establish the model, and all the indexes of the rats were in line with the characteristics of D-IBS [3, 9], indicating the success of the model. Intervention of QingHuaZhiXie prescription could improve the symptoms of diarrhea and intestinal hypersensitivity in rats, reflecting its good therapeutic effect on D-IBS symptoms.

Many inflammatory cytokines and their related signaling pathways are activated during stress response, resulting in increased intestinal permeability or visceral hypersensitivity and eventually leading to D-IBS symptoms [23, 24]. This study found that the transcription and translation levels of TLR4 were activated by D-IBS, and the expression was significantly increased. But the expression level of TLR4 was effectively inhibited after QingHuaZhiXie prescription treatment, which indicated that QingHuaZhiXie prescription could alleviate the symptoms of D-IBS. At the same time, this study also found that the remission effect of QingHuaZhiXie prescription on D-IBS was positively correlated with its dosage, that is, with the increase of dosage, its remission effect was also significantly improved. Both of the MyD88-dependent pathway and NF-*κ*B independent pathway play a pivotal role in TLR4 signal transduction. Meanwhile, NF-*κ*B plays an important role in a variety of stress diseases, such as neurodegenerative diseases, as a key regulatory factor through dynamic nuclear DNA/protein binding [25, 26]. This study found that the expression levels of MyD88 and NF-*κ*B in the QingHuaZhiXie prescription group were significantly lower than those in the D-IBS group, indicating that QingHuaZhiXie prescription can act on the two signal transduction pathways of TLR4 at the same time, thus preventing the subsequent inflammatory reaction. In the high dosage group of QingHuaZhiXie prescription, the protein expression of this pathway did not reach the level of the control group, but in the physiological level, it has basically completely relieved the disease of rats. At the same time, from the perspective of balancing the expression level of intracellular inflammatory factors, the good effect of QingHuaZhiXie prescription was also reflected. The expression level of inflammatory factors in the high-dose group is basically the same as that in the control group. Accordingly, we also found that QingHuaZhiXie prescription could reduce the MPO activity, indicating that the inflammation was relieved.

Tight junction (TJ) is an important part of intestinal epithelial cell barrier [27]. Transmembrane proteins (occluding and claudins), junctional adhesion molecules, and cytoplasmic adhesion proteins (ZOs, 7H6, and AF6) are essential to maintain the integrity of TJ [27–29]. Inflammatory factors such as IFN-*γ* and TNF-*α* can lead to the abnormal distribution of occludin protein, resulting in the disruption of TJ [30, 31]. One of the important characteristics of human intestinal inflammation is abnormal mucosal barrier function. D-IBS is closely related to the change of tight junction permeability in intestinal epithelium [31]. In D-IBS rats, the expression of intestinal mucosal marker protein decreased, the permeability increased, and the proinflammatory substances such as endotoxin in intestinal cavity entered the lamina propria to induce immune response, and the content of proinflammatory factors increased. Inflammatory cytokines such as TNF-*α* can induce epithelial apoptosis and increase intestinal permeability and visceral sensitivity [32, 33].

After treatment with QingHuaZhiXie prescription, the inflammatory response of IBS-D rats was significantly reduced, the expression of intestinal mucosal barrier marker protein was upregulated, and visceral sensitivity and gastrointestinal dysfunction were significantly improved. It is suggested that QingHuaZhiXie prescription can protect intestinal mucosal barrier by regulating the expression of occludin, claudin-1, ZO-1, and JAM in colon tissue. By inhibiting the TLR4/MyD88/NF-*κ*B pathway, QingHuaZhiXie prescription adjusts the imbalance of inflammatory factor expression and inhibits inflammatory response, which contributes to improving gastrointestinal function to achieve the purpose of treatment of IBS-D.

Chinese herbal compound prescription has become a new trend in the treatment of D-IBS because of its advantages of multicomponent and multitarget with little side effect. However, traditional Chinese Medicine formulation is a complex system with multiple components, multiple targets, and synergistic interactions among its components [34]. Because of its complex chemical composition, it is extremely difficult to study its role in the body as a mixture [35]. The complexity of TCM formulations makes their in-depth study difficult. In this study, we speculated that Radix Paeoniae Alba and Fangfeng substances of QingHuaZhiXie prescription may play important roles in the regulation of the TLR4/MyD88/NF-*κ*B signaling pathway. In any case, in the further study, we will use systems pharmacology and network pharmacology to further elucidate the molecular mechanism of QingHuaZhiXie prescription in D-IBS.

In conclusion, the positive effect of TCM formulation, QingHuaZhiXie, in the treatment of D-IBS was confirmed in this study. Depth analysis revealed that QingHuaZhiXie prescription reversed the imbalance of cytokines by acting on the TLR4/MyD88/NF-*κ*B pathway, contributing to release D-IBS symptoms.

## Figures and Tables

**Figure 1:** QingHuaZhiXie prescription treatment relieving D-IBS symptoms. (a) Abdominal withdrawal reaction (AWR) analysis. (b) Effect of QingHuaZhiXie prescription on histopathological changes in the distal colon. The middle part of distal colons was sectioned and stained with hematoxylin and eosin (H&E). ^∗∗^*P* < 0.01 and ^∗∗∗^*P* < 0.001 vs. the control group; ^#^*P* < 0.05 and ^##^*P* < 0.01 vs. the model group.

**Figure 2:** Expression levels of occludin, claudin-1, ZO-1, and JAM in six groups. The expression of occludin-1, claudin-1, ZO-1, and JAM were detected by Western blot, and *β*-actin was used as internal standard. ^∗∗∗^*P* < 0.001 vs. the control group; ^#^*P* < 0.05, ^##^*P* < 0.01, ^###^*P* < 0.001 vs. the model group.

**Figure 3:** Effect of QingHuaZhiXie prescription on TLR4/MyD88/NF-*κ*B pathway proteins expression. (a) Transcription levels of TLR4, MyD88, and NF-*κ*B. (b) Protein expression levels of TLR4, MyD88, and NF-*κ*B. ^∗∗∗^*P* < 0.001 vs. the control group; ^#^*P* < 0.05, ^##^*P* < 0.01, and ^###^*P* < 0.001 vs. the model group.

**Figure 4:** Effect of QingHuaZhiXie prescription on expression level of inflammatory factors and MPO activity. (a) Transcription levels of TNF-*α* and IFN-*γ* based on RT-qPCR analysis. (b) Expression levels of TNF-*α* and IFN-*γ* based on ELISA analysis. (c) Examined MPO activity through immunohistochemical analysis. ^∗∗∗^*P* < 0.001 vs. the control group; ^#^*P* < 0.05, ^##^*P* < 0.01, and ^###^*P* < 0.001 vs. the model group.

**Table 1:** Primers used in this study.

Gene	Forward primer (5′-3′)	Reverse primer (5′-3′)
TLR4	GGGCCTAAACCCAGTCTGTTTG	CTTCTGCCCGGTAAGGTCCA
MyD88	AAGATGACCCTGGGAGCCCTA	CTCAGGCCAGTCATCATTGAACA
NF-*κ*B	ACCACTGCTCAGGTCCACTGTC	GCTGTCACTATCCCGGAGTTCA
TNF-*α*	CTCAAGCCCTGGTATGAGCC	GGGAACAGTCTGGGAAGCTC
IFN-*γ*	GGCAAAAGGACGGTAACACG	CGAACTTGGCGATGCTCATG
*β*-Actin	GAGGGAAATCGTGCGTGAC	CTGGAAGGTGGACAGTGAG

## Data Availability

The datasets used and/or analyzed during the current study are available from the corresponding author upon request.
